# Cirrhotic cardiomyopathy: the liver affects the heart

**DOI:** 10.1590/1414-431X20187809

**Published:** 2019-02-14

**Authors:** M.V.H. Carvalho, P.C. Kroll, R.T.M. Kroll, V.N. Carvalho

**Affiliations:** 1 Departamento de Cirurgia, Faculdade de Medicina de Jundiaí, Jundiaí, SP, Brasil; 2 Hospital de Transplante E.J. Zerbini, São Paulo, SP, Brasil; 3 Instituto Dante Pazzanese de Cardiologia, São Paulo, SP, Brasil; 4 Hospital Municipal Dr. Mario Gatti, Campinas, SP, Brasil

**Keywords:** Cirrhotic cardiomyopathy, Cirrhosis, Heart failure, Cardiac cirrhosis, Hyperdynamic circulation

## Abstract

Cirrhotic cardiomyopathy historically has been confused as alcoholic cardiomyopathy. The key points for diagnosis of cirrhotic cardiomyopathy have been well explained, however this entity was neglected for a long time. Nowadays the diagnosis of this entity has become important because it is a factor that contributes significantly to morbidity-mortality in cirrhotic patients. Characteristics of cirrhotic cardiomyopathy are a hyperdynamic circulatory state, altered diastolic relaxation, impaired contractility, and electrophysiological abnormalities, particularity QT interval prolongation. The pathogenesis includes impaired function of beta-receptors, altered transmembrane currents and overproduction of cardiodepressant factors, such as nitric oxide, cytokines and endogenous cannabinoids. In addition to physical signs of hyperdynamic state and heart failure under stress conditions, the diagnosis can be done with dosage of serum markers, electrocardiography, echocardiography and magnetic resonance. The treatment is mainly supportive, but orthotopic liver transplantation appears to improve this condition although the prognosis of liver transplantation in patients with cirrhotic cardiomyopathy is uncertain.

## Introduction

For many years, cardiac dysfunctions associated with liver cirrhosis were attributed to the direct toxic effects of alcohol on the heart. However, in 1953, Kowalski and Abelmann (1) showed the existence of a circulatory dysfunction specific to liver cirrhosis. Since then, several studies have consistently reproduced those findings (2 [Bibr B03]–5). Successive publications of experimental and clinical studies have established the idea that cirrhotic cardiomyopathy (CCM) is a clinical entity different from that seen in alcoholic heart muscle disease.

Interference of liver disease with the cardiac and circulatory performance would be expected, considering that the liver receives 25% of the cardiac output. The term CCM was introduced more than three decades ago to describe a spectrum of chronic cardiac dysfunction in cirrhotic patients in the absence of known heart disease, regardless of the etiology of cirrhosis (4,6).

Hepatic cirrhosis leads to a hyperdynamic circulatory state, which induces cardiac dysfunctions that characterize the CCM syndrome. This syndrome includes, in addition to the hyperdynamic circulation, a combination of systolic (7) and diastolic dysfunctions (8–11), prolonged ventricular repolarization (12), and inability of the sinus node to increase heart rate (HR) during exercise (13).

### Epidemiology and natural history

CCM is a condition easily tolerated, remaining asymptomatic for months to years because of the near-normal cardiac function at rest, manifesting only under conditions of physical or pharmacological stress. Therefore, the diagnosis of CCM is difficult and the exact prevalence of this condition remains unknown (7).

However, it has been estimated that 40–50% of patients who underwent liver transplantation have some signs of cardiac dysfunction, which means that these patients underwent surgery under a condition of CCM (7,11,14). Furthermore, since diagnosis of CCM is frequently missed or delayed, its natural history is unclear in terms of response to treatment and prognosis (7).

As CCM is a relatively recent entity, the purpose of this review is to provide an explanation about its definition. Its pathophysiological mechanisms, criteria, and supplemental exams for its diagnosis are also included to show CCM relevance. Although the treatment of this condition is mainly supportive, the actions that should be taken to approach CCM are also commented.

## Material and Methods

Structured medical subject headings (MeSH) were used to search original articles and reviews about CCM in MEDLINE by means of the PubMed database. The term "cirrhotic cardiomyopathy" was used. A total of 275 complete articles, published until March 2018, were identified. All articles selected in the search were in English, and abstracts for oral presentations and letters to the editor were ignored. We also searched for further relevant articles in the reference lists of articles. First, titles and abstracts were read to know whether they fit the purpose of reviewing the issue. If their eligibility remained unclear, the full-text reports were then considered. Ninety studies were selected and organized to provide the authors of the present study with the means to write a narrative review including history, definition, epidemiologic data, clinical findings, diagnosis, and treatment.

## Definition of CCM

A consensus diagnostic criterion for CCM (Table 1) was established at the World Congress of Gastroenterology held in Montreal in 2005 (10). Thus, CCM is defined as a cardiac dysfunction in patients with cirrhosis, which is characterized by impaired contractile responsiveness to stress and/or altered diastolic relaxation, with electrophysiological abnormalities, in the absence of other known cardiac disorder (9,10).

**Table 1:** Proposal of diagnostic criteria for cirrhotic cardiomyopathy agreed upon at the 2005 World Congress of Gastroenterology in Montreal (10). There are suggestions (not included in this table) to improve these criteria considering dysfunction of right ventricle (15), biventricular diastolic dysfunction at rest, large left and right atria, higher systolic pulmonary arterial pressure and left ventricular mass (16) and evaluate systolic function assessment using tissue strain imaging (17).

Systolic dysfunction	Resting ejection fraction <55% Blunted increase in cardiac output with exercise or pharmacological stimuli
Diastolic dysfunction	Early diastolic atrial filling ratio (E/A ratio) <1.0 (age corrected) Deceleration time (DT) >200 ms Prolonged isovolumetric relaxation time >80 ms
Supportive criteria	Electrophysiological abnormalities (prolongation of QT) Abnormal chronotropic response Electromechanical uncoupling Enlarged left atrium Increased myocardial mass Increased brain natriuretic peptide and pro-peptide Increased troponin I

References

10. Wiese et al. doi: 10.1038/nrgastr.2013.210.

15. Chen Y et al. doi: 10.1016/j.jjcc.2015.08.001.

16. Rimbas RC et al. doi: 10.1016/j.ultrasmedbio.2017.11.013.

17. Farr M and Schulze PC. doi: 10.4137/CMC.S15722.

These diagnostic criteria are still in use. However, suggestions have been made to improve these criteria by including the dysfunction of the right ventricle as an important parameter of cardiac damage caused by cirrhosis (15). Tissue Doppler and speckle tracking imaging have also shown that CCM patients have biventricular diastolic dysfunction at rest, larger left and right atria, and higher systolic pulmonary arterial pressure and left ventricular mass (16). In addition, the systolic function assessment using tissue strain imaging is more sensitive than the usual echocardiographic indices (17).

Because alcoholism is the leading cause of hepatic cirrhosis, it is important not to confuse CCM with alcoholic cardiomyopathy, whose underlying mechanisms responsible for structural and functional cardiac abnormalities are pathophysiologically and clinically different (18). The main mechanism responsible for alcoholic cardiomyopathy is the reduction in arterial perfusion of the whole organism, which leads to hypoxia and passive venous congestion secondary to increased systemic venous pressure (19).

## Pathophysiological mechanisms

Although the major circulatory changes that lead to CCM were indicated more than half a century ago, these mechanisms have been more clearly understood only recently. Figure 1 shows a summary of the mechanisms involved in the genesis of CCM hyperdynamic circulation.

**Figure 1.** Schematic representation of the pathophysiological mechanisms that lead to liver disease to affect the heart. CO: cardiac output; HR: heart rate; AP: arterial pressure; SVR: systemic vascular resistance.

Portal hypertension leads to a state of peripheral vasodilatation due to a release of vasodilator mediators such as nitric oxide (NO), carbon monoxide, and prostacyclin (20 [Bibr B21]–22).

Progressive hepatic decompensation results in blood volume redistribution, with increased splanchnic blood flow and relatively decreased central circulation. The baroreceptors may be deactivated to compensate for the reduction in the central and arterial blood flow, with increased sympathetic nervous activity and consequent increase in HR and cardiac output (CO) (23). Therefore, hyperdynamic circulation in cirrhosis is an appropriate initial response to the splanchnic arterial vasodilation (24).

Patients with advanced cirrhosis exhibit hyperdynamic circulation with increased CO. This hyperdynamic state arises from a marked splanchnic arterial vasodilation and reduced systemic vascular resistance (25). Increase in vasodilation due to portosystemic shunting and bacterial translocation increase the hyperdynamic circulation and central hypovolemia (26).

At rest, the intra-cardiac pressures are normal because the reduced afterload secondary to the systemic vasodilation compensates for both preload reduction and contractile dysfunction. This circulatory state, which resembles those of high CO, results from increased blood flow and is defined as heart failure due to volume overload. Thus, the hyperdynamic circulation in cirrhosis is secondary to the low systemic vascular resistance and increased arterial compliance (27 [Bibr B28]–30).

## Systolic dysfunction

Several studies have shown that the left ventricular ejection fraction is normal at rest (25,30). Nevertheless, the ventricular ejection fraction after exercise increases significantly less than in non-cirrhotic patients (31,32). The aerobic exercise capacity and maximal HR in cirrhotic patients are lower than in normal subjects. This reduced cardiac performance is due to the direct low HR response to exercise (33), decreased myocardial contractility, and marked weakening and loss of the skeletal musculature, thus causing impaired extraction of and demand for peripheral oxygen (34). Systolic incompetence has been evidenced by physical and pharmacological stress tests (9). The mechanism is related to the myocardial low response in the downregulation of beta-adrenergic receptors in cardiomyocyte membranes (35).

Other inhibitory pathways contribute to decrease the cardiomyocyte contractility and, hence, decrease the systolic function in cirrhosis. Usually, the cannabinoid signaling system is minimally expressed in healthy individuals. However, a significant upregulation of the cannabinoid signaling pathway is observed in patients with cirrhosis (36). In addition, increase in the activity of inducible NO synthase and heme oxygenase promotes the production of NO and carbon monoxide, respectively, and these evanescent gases have a negative effect on cardiomyocyte contraction. Stimulation of the NO pathway is possibly related to the increased activity of cytokines in cirrhosis, as it was observed in the experimental model of cirrhotic rats (37). Furthermore, bacterial lipopolysaccharides that permeate the gut barrier enter into circulation and activate monocytes and lymphocytes to release various cytokines (30).

In summary, various studies have shown that the left ventricular ejection fraction is usually normal in patients with chronic liver disease who are at rest. In this condition, the reduced afterload, which is secondary to systemic vasodilation, compensates the preload reduction and contractile dysfunction. However, systolic dysfunction is unmasked under stress situations. Thus, cirrhotic cardiomyopathy is characterized by normal or high cardiac output. However, systolic dysfunction occurs when the heart is challenged. In such condition, the heart is unable to maintain adequate arterial circulation.

## Diastolic dysfunction

Diastolic dysfunction is characterized by a decreased rate of left ventricular relaxation, restricted blood flow into the ventricle, and increased end-diastolic pressure. According to Glenn et al. (38), alteration of titin protein modulation and collagen configuration have a role in the pathogenesis of diastolic dysfunction in cirrhosis. Titin protein is a sarcomere protein that directly influences the ventricular stiffness and diastolic function. In addition, some studies indicate that sodium and fluid retention in cirrhosis may play a role in the development of diastolic dysfunction (39 [Bibr B40]–41).

Prevalence and extent of systolic dysfunction in cirrhotic patients is variable whereas various elements of diastolic dysfunction are more frequent (42). Other authors have pointed out that some degree of diastolic dysfunction is present in all patients (8,10). Unlike systolic dysfunction, which appears in stress conditions, diastolic dysfunction can be easily seen in the echocardiography exam at rest (42,43).

In the World Congress of Gastroenterology 2005 (10), however, some criticism was directed at the criteria in relation to the transmitral flow velocities calculated using conventional pulse-wave Doppler echocardiography. That was because transmitral velocities calculated using a conventional pulse-wave Doppler have neither sensitivity nor specificity for diagnosis and grading severity of diastolic dysfunction (44).

Thus, tissue Doppler imaging could be considered to quantify left ventricular diastolic function (18). Speckle tracking is a new echocardiography technique that can offer a detailed analysis of ventricular function. It allows frame-to-frame tracking of myocardial tissue in the longitudinal, radial, and circumferential directions, providing a detailed analysis of left ventricular function (45).

Cirrhotic patients primarily manifest diastolic dysfunction with normal systolic function at rest (43). In cirrhosis, diastolic dysfunction derives from myocardial wall thickening, which is caused by left ventricular hypertrophy, altered collagen structure, fibrosis, and subendothelial edema, resulting in high left ventricular filling pressures (8,10,46). In a study with cirrhotic patients, Wong et al. (47) reported that diastolic dysfunction is of marked and decisive importance in CCM, and diastolic dysfunction affects at least 50% of patients with cirrhosis. Doppler imaging studies have shown correlation between diastolic and circulatory dysfunctions, development of ascites, hepatorenal syndrome, and survival (48 [Bibr B49]–50).

## Electrocardiographic abnormalities and chronotropic incompetence

Prolonged QT interval is the most common electrophysiological alteration, occurring in more than 50% of cirrhotic patients (51,52). This abnormality can affect the heart rhythm causing serious arrhythmias, including ventricular arrhythmia and sudden death (53).

Loss and/or dysfunction of the membrane potassium channels play a role in delayed ventricular repolarization, which may lead to QT interval prolongation (54). However, the pathophysiology of QT interval prolongation in cirrhosis has not yet been fully elucidated (55,56). Certainly, exposure of the heart to cardiotoxins such as endotoxins, cytokines, and bile salts also plays an important role in increasing the sympathetic-adrenergic tone that characterizes cirrhosis (57,58). The QT interval prolongation surely also results from hyperactivity of the sympathetic-adrenergic discharges, since excessive release of noradrenaline causes myocardial damage and beta-adrenergic receptor downregulation (59). A study showed that, in cirrhotic patients, duration of ventricular repolarization (represented by the QT interval) varies in response to minimal changes in portal pressure (58).

Chronotropic incompetence is the inability of the sinus node to increase HR after exercise or pharmacological stimulation. In CCM and under stress conditions, the sympathetic nervous system is not able to respond with adequate acceleration of the atrial and ventricular rate (60). The mechanism of this autonomic dysfunction is probably a direct inhibition of the beta-receptor mediated stimulation (61).

## Diagnosis of CCM

CCM is a relatively silent condition under stable situations. Peripheral vasodilation protects the heart by reducing the afterload and heart failure does not appear at rest. In patients suffering from cirrhosis, with intolerance to exercise and without underlying known cardiac disease, CCM should be suspected.

Although new exams are improving diagnosis accuracy, echocardiogram and electrocardiogram are essential exams to diagnose this condition.

### Electrocardiogram

Prolongation of the QTc interval (>440 ms) can be observed in cases of portal hypertension with or without cirrhosis. The frequency of QT prolongation in cirrhotic patients is in the range of 30–60% and positively correlates with the severity of liver disease (62,63).

As heart rate affects the length of the QT interval, its correction by the heart rate is always necessary. Thus, applying the Fridericia’ formula instead of the Bazett formula is preferable as the latter incompletely suppresses the relationship between QT and heart rate (64).

### Echocardiography

Echocardiography is essential in all patients with suspicion of CCM. In contrast with systolic dysfunction, diastolic dysfunction is a prominent characteristic of CCM and seems to be its first manifestation (65). In addition, diastolic impairment may affect the prognosis of cirrhotic patients regardless if liver was transplanted or not (48). The most frequent echocardiography abnormality is first-degree diastolic dysfunction. It is characterized by reduced early diastolic ventricular filling and increased atrial filling (E/A<1.0), deceleration time >200 ms, and prolonged isovolumetric relaxation time (ITVR >80 ms), which represent increased resistance to ventricular inflow (66).

Stress echocardiography is a method that should be used in patients with advanced liver disease as it can detect subtle systolic and diastolic dysfunctions before the ventricular ejection fraction is decreased. This stress test should be considered in the diagnostic approach to CCM to avoid under-diagnosis (67).

### Cardiac troponin

The structural protein troponin is a specific marker of myocardial lesion. Troponin I is a thin filament of cardiac muscle protein, which is a marker of cardiac lesions. The levels of such marker are elevated in patients with ischemia. Patients with liver cirrhosis can present high levels of troponin I (68,69).

### Cardiac biomarkers (ANP and BNP)

The atrial natriuretic peptide (ANP) is secreted in response to volumetric atrial distention, as a result of atrial overload and ventricular hypertrophy in cirrhotic patients. As patients with uncompensated cirrhosis usually exhibit changes in volume and cardiac pressures, the ANP is frequently elevated in these cases (70).

The brain natriuretic peptide (BNP) and its pro-hormones are also produced by the ventricles as a consequence of volume overload, increase in ventricular pressure, and ischemia (71). BNP and its pro-hormones are usually elevated in patients with cirrhosis (72), and BNP is considered an early marker in CCM (73).

Supplemental exams, which can contribute to the diagnosis of CCM, are presented below.

### Cardiovascular magnetic resonance (MR)

Until now, MR is considered the best exam to study heart morphology. In addition, MR with gadolinium contrast can be used to determine the chamber volumes, ejection fraction, and possible fibrosis and edema (11). The MR imaging areas of high signal intensity, which appear 10–15 min after injection of gadolinium (intracellular contrast agent) in regions of myocardial scarring, were described as late gadolinium enhancement. In case of CCM, late gadolinium enhancement has a diffuse myocardial distribution in MR images with the appearance of myocarditis (74,75). Furthermore, MR images can indicate an impaired cardiac response under pharmacological stress testing with dobutamine. Deformation analysis parameters of MR images may be more sensitive than conventional methods in identifying abnormalities in the inotropic response to stress (76).

## Controversial issues

In patients with liver cirrhosis, cardiac dysfunction may be related to arterial hypertension and ischemic and alcoholic heart disease. Hepatic disease may likewise cause anemia, which also affects cardiac structure and function. Therefore, the relationship between cirrhosis and cardiac disease cannot be assured (77).

## Treatment of CCM

CCM is a clinically silent or mild entity, and symptoms of heart failure become evident when stress occurs. Thus, there is little interest or necessity in treating CCM at the asymptomatic stage. As far as is known, there is no clinical study on the management of CCM. When some form of stress occurs, and heart failure clinically manifests, the guidelines for the treatment of chronic heart failure in non-cirrhotic patients can be followed. However, in advanced phases of cirrhosis, reduction in cardiac afterload is not recommended, as these patients are already significantly vasodilated (78).

Liver transplantation can be a definitive treatment for patients with cirrhosis, but the unavailability of organ donors and cost concerns should be considered. The candidates must be well evaluated, as patients are at risk of death by heart failure, coronary artery disease, tachyarrhythmias, and other cardiac deaths in the post-operative term of liver transplantation. Thus, there are no accurate data on prognosis for liver transplantation in patients with CCM. However, diastolic dysfunction significantly worsens after transplantation in these patients (79).

Patients with CCM should be recommended to avoid physical effort and other forms of stress, and oxygen should be provided in some situations. Medications can have adverse effects or weak response in patients with CCM, and specific pharmacological treatment with proven efficacy in CCM is not currently available now. However, when some form of stress occurs and heart failure becomes evident, the guidelines for treatment of chronic heart failure can be followed at least in the pre-ascites phase.

Non-selective beta-blockers have shown to reduce the prolonged QT interval and might reduce the hyperdynamic load in patients with cirrhosis, but whether the correction of QT interval has a positive effect on prognosis is doubtful (80). In addition, the use of beta-blocker drugs by patients with refractory ascites has a risk of increased mortality (81). Furthermore, patients with cirrhosis cardiomyopathy received a six-month therapy with metoprolol, and beta-blockage with this drug did not improve heart function and morphology (82).

In a revision of 10 hemodynamic studies on liver cirrhosis, Tripathi and Hayes (83) concluded that carvedilol is a potent agent to reduce portal pressure. However, careful dosing is necessary to minimize adverse effects, especially reduction in the mean arterial pressure. Doses as low as 12.5 mg have shown an efficacy that is similar to that of higher doses, and probably represent the best compromise between efficacy and side effects.

Angiotensin converting enzyme inhibitors can improve diastolic function in patients with cirrhosis by decreasing the ventricular thickness and dilation, but they should be used in the early phases of cirrhosis because of the risk of hypotension and hepatic-renal syndrome in later phases (84). Even though these drugs reduce the portal pressure in patients with cirrhosis, they should be discontinued if ascites appears, as they can further aggravate the systemic vasodilation state and increase the risk of hepatorenal syndrome (18,85).

Spironolactone is a competitive aldosterone inhibitor and should be used as a diuretic in patients with severe heart failure as it has been shown to reduce the frequency of hospitalization and mortality (86). In addition, aldosterone receptor antagonists seem to reduce the hepatic-venous pressure gradient, the ventricular wall thickness, and the left ventricular end-diastolic volume (86,87).

Liver transplant is the only effective treatment established for patients with final stage liver disease associated with CCM. Liver transplantation has been shown to reverse the systolic and diastolic dysfunction and prolonged QT interval (88).

However, many cardiac complications and some cardiac deaths have been reported in patients undergoing liver transplantation. This fact can be attributed to cardiac dysfunction due to previous CCM (89).

Unfortunately, no reliable method to identify patients susceptible to develop perioperative cardiac complications is currently available (29).

## Conclusions

Liver cirrhosis can induce cardiac abnormalities characterized by an impaired stress response, diastolic dysfunction, and electrocardiographic changes (CCM). No symptom is seen at rest, but heart failure can be unmasked under stress conditions. This occurs because at rest the diastolic and systolic dysfunctions are counterbalanced by the specific hyperdynamic state of cirrhosis. Pathogenesis of CCM includes mechanisms such as increased activity of the vasodilator pathway through the actions of NO, carbon monoxide, cytokines, and cannabinoids, decreased beta-adrenergic function, and sodium and calcium transport kinetics downregulation in the cardiac muscle, leading to an impaired contractile function of the cardiomyocyte. Echocardiogram and the electrocardiogram are the most important exams for diagnosis of CCM, but cardiac magnetic resonance imaging and biomarkers are currently becoming more relevant than before.

The treatment of CCM is directed to left ventricular failure, with sodium restriction, diuretics, and afterload reduction. Liver transplantation may improve or normalize cardiac function.
